The article "Automatic neonatal sleep stage classification: A comparative study" was published in 2023. Journal: Heliyon.

# Automatic neonatal sleep stage classification: A comparative study

**DOI:** 10.1016/j.heliyon.2023.e22195

**Published:** 2023-11-13

**Authors:** Saadullah Farooq Abbasi, Awais Abbas, Iftikhar Ahmad, Mohammed S. Alshehri, Sultan Almakdi, Yazeed Yasin Ghadi, Jawad Ahmad

**Affiliations:** a Department of Electronic, Electrical and System Engineering, University of Birmingham, Birmingham, United Kingdom; b James Watt School of Engineering, University of Glasgow, United Kingdom; c Department of Computer Science, College of Computer Science and Information Systems, Najran University, Najran, Saudi Arabia; d Department of Computer Science, Al Ain University, Abu Dhabi P.O. Box 112612, United Arab Emirates; e School of Computing, Engineering and the Built Environment, Edinburgh Napier University, Edinburgh EH10 5DT, UK

**Keywords:** Neonatal sleep staging, Polysomnography, Classification, Electroencephalography

## Abstract

Sleep is an essential feature of living beings. For neonates, it is vital for their mental and physical development. Sleep stage cycling is an important parameter to assess neonatal brain and physical development. Therefore, it is crucial to administer newborn's sleep in the neonatal intensive care unit (NICU). Currently, Polysomnography (PSG) is used as a gold standard method for classifying neonatal sleep patterns, but it is expensive and requires a lot of human involvement. Over the last two decades, multiple researchers are working on automatic sleep stage classification algorithms using electroencephalography (EEG), electrocardiography (ECG), and video. In this study, we present a comprehensive review of existing algorithms for neonatal sleep, their limitations and future recommendations. Additionally, a brief comparison of the extracted features, classification algorithms and evaluation parameters is reported in the proposed study.

## 1 Introduction

Sleep is a complex physiological state that involves orchestrated changes in brain activity, muscular relaxation, and alterations in sensory responsiveness. It is a fundamental process essential for maintaining both mental and physical well-being. Sleep serves various crucial functions, including energy conservation, consolidation of neural connections, memory processing, and facilitation of mental and physical development, particularly in neonates. Monitoring neonatal sleep patterns through intensive neuro-monitoring at the bedside allows for a comprehensive understanding of normal neurological function [[1], [2], [3]].

Neonatal sleep measurement holds paramount clinical importance for paediatricians and neonatologists. Administration and maintenance of newborns require a detailed assessment and deep understanding of neonatal sleep patterns. These patterns help paediatricians to supervise and monitor the progress in growth and health of newborns. Correlation between sleep cycle and brain development is of essential significance, therefore, observation and evaluation of sleep patterns and their time span in infants reflect the functioning and overall wellness of neonatal brains.

The article "Automatic neonatal sleep stage classification: A comparative study" was published in 2023. Journal: Heliyon.

This precise evaluation of sleep patterns can play a vital role in the early diagnosis of sleep disorders in infants. These disorders can hinder the brain development, consequently causing health issues. However, early diagnosis of sleep disorders like sleep apnea or movement disorders during sleep can be made by coherent analysis of sleep cycles. This can help health professionals to take timely and appropriate measurements for improving neonatal health. These measures also lead to asses the effectiveness of healthcare interventions and treatment therapies targeting sleep quality elevation and nurture healthy maturation. Ultimately, better healthcare plans for infants can be devised. Analysis of sleep patterns in new borns can also provide valuable insights for the functioning of metabolism and immune system due to the connection between sleep and physiological processes. These insights can lead to advancements in neonatal healthcare.

There are two major methods used for recording an infant's sleep: polysomnography (PSG) and behavioral sleep measurement. Notably, research on both approaches has identified certain limitations [4]. Classification of sleep stages can be achieved using three methods: utilizing PSG technique alone [[5], [6], [7], [8], [9]], employing behavioral approaches [[10], [11], [12], [13]], or combining both methods simultaneously [[14], [15], [16], [17], [18]]. The standard procedure for classifying an infant's sleep pattern typically involves the manual interpretation of EEG pointers. Accurate sleep recording is a crucial aspect of this process, essential for reaching accurate diagnoses and determining appropriate treatments, which are grounded in various biological accounts. Although the conventional visual scoring technique involves interpreting diverse indicators or signals, it is considered the most widely accepted method [19]. However, the qualitative nature of scoring can lead to variations in results among different experts due to differences in experience [20,21].

Optimistically, when two experts agree on the obtained results and conclusions, the average agreement ratio is approximately 83 ± 3 % [22], which may not be entirely convincing. Additionally, visual examination based on EEG labelling for the entire night can be time-consuming. Therefore, the use of an automatic recording process is deemed a well-organized method [23,24]. Sleep consists of two major stages: Non-Rapid Eye Movement (NREM) and Rapid Eye Movement (REM) sleep. Active Sleep (AS), also known as REM sleep, occurs in intervals of 5–30 min with 70-min intervals. Neural activity during REM sleep is significantly higher compared to NREM sleep. In contrast, during NREM sleep, or Quiet Sleep (QS), blood pressure, metabolic rate, heart rate, and sympathetic activity decrease, while parasympathetic activity increases. Sleep specialists typically adhere to firm guiding principles for sleep scoring, which are based on strategies established by standardization bodies [25,26]. In Fig. 1, the time consumed in every sleep phase over the whole period of neonatal age is given [27].

The article "Automatic neonatal sleep stage classification: A comparative study" was published in 2023. Journal: Heliyon.

**Fig. 1:** Percentage of QS and AS with respect to gestational age [27].

Numerous researchers have recently proposed various approaches to systematize the procedure of sleep classification, commonly known as sleep scoring. Signal processing methods and machine learning techniques have been extensively explored to derive valuable insights from biological signals [28]. However, when it comes to neonatal sleep staging, the utilization of certain features and classifiers has yielded limited success due to technological challenges. Many of these approaches have relied on characteristics typically employed in adult sleep research, such as time and frequency domains, as well as nonlinear and complexity aspects [29]. Consequently, these techniques are often applied to conflicting types of sleep classification. Notably, the neonatal sleep stage classification algorithm can be categorized into four types: quiet sleep detection, sleep-wake classification, three-stage classification, and tetrad stage classification [30,29,31]. Later in this study, we will delve into the details of these algorithms, including the data used and their outcomes.

Our study establishes that specific physiological indicators contain valuable information regarding sleep phases. These facts and figures are further employed to support analysis, treatment observation, and assessments of drug effectiveness. The extraction of information and the measurement of signals are crucial for harnessing the benefits mentioned. However, there is currently no standardized procedure for extracting information from physiological signals, leading to ambiguity in determining which signal provides sufficient evidence for accurate diagnosis.

To address this ambiguity, we have revised the mechanisms for extracting material from altered physiological signals, aiming to provide a signal that is essentially data-driven. Recognizing the significance of automatic sleep phase scoring in future work, we emphasize the role of computer machinery in reducing inter-observer and intra-observer inconsistencies. Integrating advanced technology with manual analysis can result in cost savings. Computer-centered systems have the potential to enhance the quality of extracted evidence by leveraging decision support classifications to assist in signal interpretation.

The article "Automatic neonatal sleep stage classification: A comparative study" was published in 2023. Journal: Heliyon.

The rest of the paper is organized as follows: Section 2 presents the methodology of the proposed review, Section 3 provides a comprehensive review of automatic neonatal sleep stage classification, exploring the existing methodologies, techniques, and algorithms employed in this field. Section 4 identify the limitations associated with current approaches to neonatal sleep stage classification. By recognizing these limitations, we aim to shed light on the areas that require further research and improvement. Section 5 focuses on future directions and potential avenues for advancement in automatic neonatal sleep stage classification. Finally, Section 6 concludes the paper by summarizing the key findings, emphasizing the clinical relevance of automatic neonatal sleep stage classification, and providing insights into the implications for pediatric practice.

## 2 Methodology

To ensure a comprehensive and systematic review, this study focused on identifying relevant studies published between 2011 and December 2022. Electronic searches were conducted in the PubMed and Web of Science databases using specific keywords related to machine/deep learning techniques and sleep scoring. The selected keywords included terms such as ‘deep learning’, ‘deep neural network’, ‘machine learning’, ‘SVM’, ‘Random Forest’, ‘convolutional neural network’, ‘recurrent neural network’, ‘CNN’, ‘RNN’, ‘LSTM’, combined with ‘neonatal sleep’, ‘neonatal sleep scoring’, ‘neonatal sleep stage’, and ‘neonatal sleep staging'.

In this research, a total of 103 records have been considered for detailed analysis. At first, 85 research articles were considered out of which 55 records were from Web of Science and 32 from PubMed. While these articles were being thoroughly studied, 18 more articles were found relevant from references, leading to a total of 103 records. In the screening phase, first and second authors followed the inclusion criteria process independently and removed duplicates. Any discrepancy was resolved through mutual consultation among all authors. This screening process lead to the selection of 25 records, taking into account the most recent addition by same team of researchers.

Following conditions were followed for including specific studies: 1) Polysomnography (PSG) data from neonatal subjects who were 37 ± 5 weeks gestational age was used; 2) Automated sleep-scoring methods were employed using only EEG signals, ECG signals, video, or a combination of these with audio signals; 3) Rules set by the American Academy of Sleep Medicine (AASM), were utilized to score the sleep states taking into account three different sleep states; 4) Use of a clinical setting or a sleep research facility for the PSG data collection; 5) Implementation of deep learning techniques directly to raw data or spectrogram images; 6) Machine learning methods were applied to specifically crafted features; 7) The study was published in English, in peer-reviewed journals or presented at scientific conferences or workshops.

The article "Automatic neonatal sleep stage classification: A comparative study" was published in 2023. Journal: Heliyon.

Out of 25 records, a total of 15 studies met the inclusion criteria for review. All of these studies comprise of machine and deep learning-based methodologies for neonatal sleep analysis, enhancing the understanding of this research area.

## 3 Automatic neonatal sleep classification

This part of the research is focused on reviewing the relevant literature on automatic sleep stage scoring. Specifically, our analysis is organized based on different physiological signals i.e. EEG and ECG. We have presented a detailed table summarizing the sleep classification results for each signal. A substantial number of systematic studies have been examined for this review. In the following subsections, we will briefly explain the neonatal sleep stage classification algorithms using different physiological signals.

### 3.1 Electroencephalography (EEG)

The electrical activity occurring in the brain is recorded through EEG. These recordings These recordings reveal distinct features during different sleep stages, which have been utilized for the development of various sleep stage classification systems [[32], [33], [34], [35]]. The first EEG of humans was recorded by Hans Berger in 1924 [36]. The brain's electrical activity is captured through electrical compulsions and is measured from the scalp of the patient. Electrodes are placed according to the standard 10–20 systems for electrode placement [37]. Clear EEG patterns indicating sleep-wake cycling (SWC) can be observed by neurologists from 30 weeks' postmenstrual age [38]. In 1937, Loomis et al. emphasized the significant application of EEG-based analysis of human sleep patterns [39]. Subsequently, after the innovative research of Loomis, several methods have been proposed for adult sleep staging using machine learning [[40], [41], [42], [43]] and deep learning [[44], [45], [46], [47]]. Profound learning methods for sleep classification include convolutional neural network (CNN) [44], recurrent neural network (RNN) [45], the combination of CNN or RNN [46,47] along with Long Short-Term Memory (LSTM) [48,49].

The article "Automatic neonatal sleep stage classification: A comparative study" was published in 2023. Journal: Heliyon.

The automatic sleep stage algorithms are distributed in two major classifications: hand-crafted feature-based classification and deep learning-based classification. In the handcrafted feature extraction approach, an extensive range of signal processing methods have been used to extract sleep-correlated data from EEG signals comprising: time domain, frequency domain, and spatial domain. The classification stage encompasses various algorithms, with deep learning and machine learning being the main approaches. Table 1 Shows a comparison of the neonatal sleep phase arrangement algorithms in detail.

**Table 1:** Review/comparative analysis of neonatal sleep-stage classification.

Author	Electrophysiological Signal	Dataset	Epoch Length (sec)	Feature	Classification Type	Classification Method	Classification Results	
							Accuracy (%)	Kappa
**L**. **Fraiwan** [50]	Electroencephalography	University of Pittsburg (29 recordings)	30	Time-Frequency Analysis	Three- stage	Artificial Neural Network	84	0.65
**L**. **Fraiwan** [51]	Electroencephalography	University of Pittsburg (27 recordings)	30	Multiscale Entropy	Three- stage	Neural Networks, Random Forest	81.3	–
**Koolean** [52]	Electroencephalography	Medical University Vienna (67 recordings)	600	57 features time, frequency and spatial	QS and AS classification	Support Vector Machine	85	–
**L**. **Fraiwan** [53]	Electroencephalography	University of Pittsburg (29 recordings)	60	7 temporal and spectral features	Three-stage	Deep Autoencoders	80.4	–
**K**. **Pillay** [30]	Electroencephalography	University Hospital of Leuven (16 recordings)	30	112 features time, frequency and spatial	2-stage classification	Hidden Markov models	95	0.89
					4-stage classification		8	0.62
**A**. **H**. **Ansari** [54]	Electroencephalography	University Hospital of Leuven (26 recordings)	30	–	QS detection	Convolutional neural network	92 AUC	0.74
**A**. **Dereymaeker** [55]	Electroencephalography	University Hospital of Leuven (26 recordings)	–	9 time and frequency domain	QS detection	CLASS	97 AUC	0.93
**H**. **Ghimatgar** [29]	Electroencephalography	University Hospital of Leuven (16 recordings)	30	–	4-stage classification	Bi-Long Short Term Memory	78.9–82.4	0.71–0.76
**A**. **H**. **Ansari** [31]	Electroencephalography	University Hospital of Leuven (42 recordings)	30	–	2-stage classification	Convolutional neural network	–	0.76
					4-stage classification			0.64
**S**. **F**. **Abbasi** [56]	Electroencephalography	Fudan University (19 recordings)	30	8-time and 4-frequency domain	Sleep-wake classification	Multi-layer perceptron	82.53	0.62
**S**. **F**. **Abbasi** [57]	Electroencephalography	Fudan University (19 recordings)	30	8-time and 4-frequency domain	Three-stage classification	Ensemble learning	81.99	–
**J**. **Werth** [58]	Electrcardiography	Philips (34 recordings)	30	–	4-stage classification	Recurrent neural network	–	0.33
**M**. **Awais** [59]	Videos	Fudan University (19 Recordings)	300	–	Sleep-wake classification	Convolutional neural network	93.8	–
**S**. **Cabon** [60]	Audio and Video	The University Hospital of Rennes	–		semi-automatic eye state estimation and sleep stage classification	5 diferent classification methods were compared.	99.4	0.5 for RF
**L**. **Fraiwan** [61]	Electroencephalography	University of Pittsburg (29 recordings)	300	–	Three stage classification	Long-short term memory	96.81	–

In the context of neonates, ECG-based neonatal sleep stage classification is very limited. For this reason, we mentioned the comparison of ECG-based neonatal sleep classification and the EEG-based classification. Table-1 Shows the comparison of the neonatal sleep stage classification algorithms in detail.

The article "Automatic neonatal sleep stage classification: A comparative study" was published in 2023. Journal: Heliyon.

### 3.2 Electrocardiography (ECG)

The electrical activity generated by the human heart is captured through the ECG signals. ECG signals exhibits a structured pattern, especially in the absence of heart disease and individual signal components can be identified through visual inspection [62]. Delicate variations in the ECG signal reflect specific sleep stages. Studies by Yucelbas et al. Xiao et al., and Kesper et al. suggest that sleep staging using ECG signals is slightly less complex but still accurate compared to PSG analysis [[63], [64], [65]]. Redmond et al. provided additional support for the rationality of ECG-based sleep staging by associating it with EEG-established sleep staging [66,67]. Fell et al. proposed the application of nonlinear examination of ECG signals for sleep staging [68,69].

### 3.3 Video-based classification

This classification involves the analysis of neonatal facial expressions to determine sleep or wake states. It is crucial to have a reliable neonatal face detection method that minimizes the inclusion of non-face-related regions, allowing for the automatic identification of sleep or wake states based on facial expressions. Recently, Awais et al. proposed a hybrid deep convolutional neural network for neonatal sleep-wake classification [59]. The algorithm utilized five deep Conv layers for automatic feature extraction, followed by classification using support vector machines. The proposed algorithm achieved an impressive accuracy of 93.8 %, which to date is the highest classification accuracy for neonatal sleep-wake classification. According to the literature, it is widely accepted that neonatal EEG can be classified as sleep when the neonate's eyes are closed. Therefore, this should be considered an important signal for automatic neonatal sleep stage classification.

The article "Automatic neonatal sleep stage classification: A comparative study" was published in 2023. Journal: Heliyon.

### 3.4 Combination

Based on our thorough research, the performance of sleep stage classification algorithm has been examined using a combination of different bio-physiological signals i.e. combination of EEG and ECG, EEG and electrooculogram (EOG), and EEG + EOG + ECG. Interestingly, in existing neonatal research, not a single algorithm has been found that utilizes a combination of multi signals for classification.

Fig. 2 shows the percentage of different bio-physiological signals employed for neonatal sleep stage classification.

**Fig. 2:** Percentage of bio-physiological signals used for neonatal sleep stage classification in existing research.

## 4 Limitations

The overall performance of the existing algorithms is commendable; however, there are still some limitations that needs to be acknowledged.

[1] Neonates are delicate and susceptible to disturbances caused by electrode placement, which can affect their sleep. For this reason, parents may feel insecure and uneasy about subjecting their child for a monitored environment. These limitations make it challenging to conduct the neonatal sleep research in an ordinary environment. However, due to the electrode placement and monitoring, this study will still need professional caretakers for data extraction. This monitored environment can only be available in the NICU. Parents usually have an increased risk of depression, anxiety, and stress after discharge from the NICU. Therefore, unless we remove 100 % human intervention, this will count as a limitation of this study.
[2] In the above table, it can be analyzed that the dataset used for neonates' sleep classification is limited. In literature, it is believed that a larger dataset yields better performance compared to a limited dataset. Therefore, acquiring larger dataset is essential for achieving better results.
[3] Existing research tends to combine amalgamates AS and wake state into low voltage irregular (LVI) signals. Corrupting overall classification authenticity. This needs to be addressed in future studies to enhance the authenticity of the classification process.

## 5 Future work

Researchers can work on several interesting ideas to improve the quality of automated neonatal sleep stage classification. The following ideas can be considered for future study.

[4] According to the AASM neonatal sleep stage classification guidelines, it is believed that a neonate is sleeping when the eyes of a neonate are closed. Therefore, in addition to EEG, EOG signals should be extracted in future studies. The classification is then done by assembling EEG and EOG features. Only two additional electrodes will be needed for this. According to my assiduous research, this ensemble can increase the accuracy of the sleep stage classification algorithm to 10–15 %. For annotation, multiple neurologists should be hired to have authentic annotation. Initially, pair of neurologists should separately annotate the sleep stages then the third neurologist will compare the annotation and make a concluding annotation based on his knowledge and existing annotation.
[5] After the situation of the global pandemic (Covid-19) will become better, there is a need to collect a larger dataset for neonatal sleep. A larger dataset will increase the accuracy of the classification network. Deep learning algorithms like CNN, RNN, and LSTM should then be applied to raw EEG data for classification. Feature extraction is a hectic process, as it is difficult to select relevant features for sleep. Therefore, in future studies, the main task is to classify sleep stages from raw EEG data. Also, at least, 3–4 sleep cycles for 1 subject should be included in the dataset. This will give a more complete dataset, as all subjects will have the same number of AS, QS, and awake epochs.
[6] Neonates are very fragile subjects and prone to these heavy and uncomfortable electrodes. Recently, multiple unobtrusive methods were published for EEG and ECG extraction. These methods should be applied in neonatal sleep. The burden of EEG electrodes can affect the sleep quality of neonates. Therefore, it is particularly important to study unobtrusive methods for automatic neonatal sleep stage classification. This unobtrusive method will help to get parental consent easily, as there is no need to attach heavy wire electrodes to the neonatal body for data extraction. Also, this will help to reduce the depression, anxiety, and stress of the subject's parents.
[7] Recently, an article has been published on neonatal sleep-wake classification using video data [59]. In the future, it will be very interesting to combine two methods i.e. sleep-wake classification using video data and QS detection using EEG. VEEG data will be extracted for this study. Then, for classification, the study will be divided into two parts. Firstly, sleep-wake segments will be separated using video data. Recently, Awais et al. published an article using neonatal video data. These sleep segments will then be used for further classification. QS can be classified with EEG with an accuracy of up to 95 %. I believe this combination can be the breakthrough for neonatal sleep stage classification soon.

The article "Automatic neonatal sleep stage classification: A comparative study" was published in 2023. Journal: Heliyon.

## 6 Conclusion

The analysis and classification of sleep stages heavily rely on physiological signals, as they provide valuable information about the different phases of sleep. Extracting and interpreting this data is the primary task of a decision support system, which then presents it to healthcare practitioners. In the context of neonatal sleep stage scoring, the focus is on utilizing physiological signals and their inherent information. In our investigation of various automated neonatal sleep stage algorithms, it became evident that EEG is the most accurate method for classifying sleep stages. However, certain stages exhibit signals that are indistinguishable from one another, necessitating the integration of multiple bio-physiological signals to improve the outcomes of the neonatal sleep stage classification algorithm. Additionally, obtaining a larger dataset is essential to achieve better results, as deep learning algorithms tend to perform more effectively when applied to extensive datasets. In conclusion, while the existing sleep stage classification algorithms have reached a mature stage, further improvements are necessary to address the identified issues and enable their full clinical utilization.

## Data availability statement

No data was used for the research described in the article.

## Funding statement

The authors are thankful to the Deanship of Scientific Research at 10.13039/501100005911Najran University for funding this work under the research groups funding program grant code (NU/RG/SERC/12/3).

## Additional information

No additional information is available for this paper.

## CRediT authorship contribution statement

**Saadullah Farooq Abbasi:** Formal analysis, Methodology, Writing – original draft, Writing – review & editing. **Awais Abbas:** Formal analysis, Methodology, Writing – original draft, Writing – review & editing. **Iftikhar Ahmad:** Formal analysis, Writing – review & editing. **Mohammed S. Alshehri:** Funding acquisition, Writing – review & editing. **Sultan Almakdi:** Formal analysis, Funding acquisition, Writing – review & editing. **Yazeed Yasin Ghadi:** Formal analysis, Writing – review & editing. **Jawad Ahmad:** Conceptualization, Funding acquisition, Methodology, Writing – review & editing.

## Declaration of competing interest

The authors declare that they have no known competing financial interests or personal relationships that could have appeared to influence the work reported in this paper.
